The article "Deepfake Video Detection Based on EfficientNet-V2 Network" was published in 2022. Journal: Comput Intell Neurosci.

# Deepfake Video Detection Based on EfficientNet-V2 Network

**DOI:** 10.1155/2022/3441549

**Published:** 2022-04-15

**Authors:** Liwei Deng, Hongfei Suo, Dongjie Li

**Affiliations:** Heilongjiang Provincial Key Laboratory of Complex Intelligent System and Integration, School of Automation, Harbin University of Science and Technology, Harbin 150080, China

## Abstract

As technology advances and society evolves, deep learning is becoming easier to operate. Many unscrupulous people are using deep learning technology to create fake pictures and fake videos that seriously endanger the stability of the country and society. Examples include faking politicians to make inappropriate statements, using face-swapping technology to spread false information, and creating fake videos to obtain money. In view of this social problem, based on the original fake face detection system, this paper proposes using a new network of EfficientNet-V2 to distinguish the authenticity of pictures and videos. Moreover, our method was used to deal with two current mainstream large-scale fake face datasets, and EfficientNet-V2 highlighted the superior performance of the new network by comparing the existing detection network with the actual training and testing results. Finally, based on improving the accuracy of the detection system in distinguishing real and fake faces, the actual pictures and videos are detected, and an excellent visualization effect is achieved.

## 1. Introduction

With the rise and development of information science, the era of deep learning has been coming. While deep learning has been a major success in computer vision, surpassing many traditional methods, over the past few years, it has been misused in the creation of fake videos, leading to a flood of fake videos on the Internet, notably artificial intelligence's deep face-swapping technology (deepfake) [1]. Deepfake technology involves altering or replacing facial information from the original video and synthesizing fake speech to create pornographic movies, fake news, political rumors, and more [2].

Accessible open-source software and apps for such face-swapping lead to large amounts of synthetically generated deepfake videos appearing in social media and news, posing a significant technical challenge for the detection and filtering of such content [3]. Since deepfake videos only need a small number of face photos to achieve video face-changing, some malicious users use the data available on the Internet to generate numerous fake videos and apply them in gray areas, such as replacing pornographic heroines with female celebrities, forging some video content for politicians, company executives, and other influential people, using synthetic fake videos to lend money to others. Thus, the purpose of misleading public opinion, winning the election, and cheating money will be achieved [4]. The content of these fake videos is extremely realistic and often accompanied by audio tampering as it is created, making it almost impossible for Internet users to identify. If these deeply falsified contents are widely disseminated through the means of the Internet, it will have a serious negative impact on the stability of the country and society [5, 6]. Furthermore, in case investigation and accident evidence collection, the lack of identification of deep fake image data will pose a huge challenge to the judicial system [7]. Thus, it is particularly important to have the ability to identify such deepfake videos and extremely urgent to perfect a systematic and efficient forged video identification system [8].

The article "Deepfake Video Detection Based on EfficientNet-V2 Network" was published in 2022. Journal: Comput Intell Neurosci.

Currently, the most commonly used deepfake face video technologies are as follows: Cycle Consistent Generative Adversarial Networks Technology (Cycle GAN) [9], that is, the source image and target image feature learning and feature conversion, but the effect is not ideal; face-changing technology (Face2Face) [10], that is, to operate on the target's facial movements and expressions with the help of the face operation database (Dlib, OpenCV), but the effect is general; deepfake technology [11], that is, the most popular and widely spread deep learning face-changing technology, which uses the neural network to learn features and then performs face synthesis. It works amazingly well, and it is difficult to distinguish the authenticity with the naked eye.

There are four types of facial manipulations that are commonly used nowadays [12]:

- *Face Attribute Manipulation*. This type of facial manipulation, also known as face editing or face retouching, uses GAN to modify some attributes of the face, such as hair, skin tone, gender, age, and adding glasses. The technology can be used to try out a variety of products, such as cosmetics, glasses, or hairstyles, in a virtual environment, allowing users to try out a variety of external modifications that suit them.
- *Face Expression Manipulation*. This type of facial manipulation, also known as facial reconstruction, allows you to freely modify a person's facial expression and even use your expression changes to control the expression changes of the subject in the video. If mishandled, facial manipulation can manipulate the facial expressions of politicians and other public figures, with serious consequences.
- *Entire Face Synthesis*. This kind of facial manipulation usually uses Cycle GAN technology to create a high-quality face that does not exist in the real world, with a high level of realism, which is difficult to distinguish with the naked eye. The technology benefits many industries such as video games and 3D modeling, but it could also be used to create fake profiles on social networks to generate dangerous industries such as misinformation.
- *Face Identify Swap*. Facial manipulation can replace one person's face in a video with another. This kind of manipulation can already be flexibly applied to many videos by most people. On the one hand, the manipulation can benefit a variety of different industries, especially the film industry. However, on the other hand, it may also be used for purposes that violate moral principles or even laws, such as celebrity pornographic videos, pranks, and financial fraud.

The article "Deepfake Video Detection Based on EfficientNet-V2 Network" was published in 2022. Journal: Comput Intell Neurosci.

In this paper, we perform efficient detection of forged video footage using deepfake technology for face identify swap. After our preprocessing, the original video-level dataset is simplified to the face image-level dataset that appears in the video, and the real face is marked as label 0 and the fake face is marked as label 1, so that the detection results of the image to be detected are displayed with a score of 0 to 1 (the closer the score is to 0, the closer the image is to the real; the closer the score is to 1, the closer the image is to fake), which greatly reduces the workload of the detection process and improves detection efficiency. The video-level datasets used in this paper are the face forensics datasets (FaceForensics++, FF++) [13], which are widely used in the detection of various fake videos, and the newly proposed and publicized face forensics datasets in the wild (Face Forensics in the Wild, FFIW_10K_) [14]. The training and evaluation of detection models are performed on these two large-scale fake face video datasets.

The detection of deepfake videos is ultimately a binary classification problem. In the preliminary investigation, we compare many efficient and excellent classification networks and finally choose the new efficient network (EfficientNet-V2) [15] as the baseline network of the detection model and optimize the network. In order to fully illustrate that the improved network is superior to other networks in all aspects, we compare the improved network with the network before improvement and other networks in terms of detection accuracy, training, and testing results. Ultimately, we confirm the efficient detection performance of this new network.

In order to enhance the visual effect of the detection system, we propose a visualization method. The image-level detection is upgraded to video-level detection, that is, after inputting the video to be detected, the video is divided into a variety of frames, and then face recognition and detection are performed on each frame (it can contain multiple faces) to select and mark the real and fake faces separately. Finally, the video frames are recombined and output to synthesize a new video, which makes the detection of fake videos more intuitive and concrete.

The article "Deepfake Video Detection Based on EfficientNet-V2 Network" was published in 2022. Journal: Comput Intell Neurosci.

The rest of the paper is structured as follows: Section 2 reports the literature review of the recent related work; Section 3 reports the preprocessing process of the dataset and the theoretical basis of the novel detection network; Section 4 collects the experimental results and shows the visualization; finally, Section 5 summarizes the full text and makes arrangements for the future work.

## 2. Related Work

As deep forgery videos have caused serious consequences to social development and network security, many related scholars have carried out a certain degree of research on this. This section mainly introduces the baseline network EfficientNet we use and briefly reviews previous work on deepfake video detection.

### 2.1. EfficientNet Network

In recent years, the convolutional neural network [16] has developed rapidly, but its deficiencies have gradually emerged. Convolutional neural networks are usually developed under a fixed resource budget. If the resources change, accordingly the network depth, network width, and input image resolution need to be manually adjusted, which brings a lot of inconvenience to scientific research. With that in mind, in 2019, Tan and Le [17] first proposed an efficient network called EfficientNet. It uses a simple and efficient compound factor to scale the network from three dimensions, network depth, network width, and input image resolution, rather than the traditional method of arbitrarily scaling the network dimensions, based on neural architecture search technology [18] to obtain the optimal set of parameters (composite coefficients). According to the degree of scaling, the EfficientNet series network can be subdivided into eight subnetworks B0–B7. After practical testing and verification, the EfficientNet network is not only much faster but also more accurate than other traditional networks.

In the subsequent research and exploration, scholars found that the EfficientNet series network could not complete the training and learning tasks excellently due to the constraints and limitations of experimental equipment after continuous practical training tests. Therefore, in 2021, Mingxing Tan et al. further improved the EfficientNet network, created a new EfficientNet-V2 network, and divided it into three subnetworks of S, M, and L. After experimental verification, compared with the old EfficientNet-V1, the new network is more streamlined, uses fewer resources, and has higher actual test accuracy.

The article "Deepfake Video Detection Based on EfficientNet-V2 Network" was published in 2022. Journal: Comput Intell Neurosci.

### 2.2. Deepfake Detection

Deep forgery videos have exploded on the Web in recent years, which has attracted widespread academic attention. Many scholars have made a detailed summary of the existing detection algorithms [12, 19, 20]. At present, part of the work of detecting deepfake videos mainly focuses on the detailed features to identify authenticity. In 2018, Li et al. [21] proposed a method based on the detection of blinking action in videos, which is a physiological signal that is not well represented in synthetic fake videos. The method works well in the benchmark test of the set and also performs well in the actual detection of deepfake generated videos. Similarly, in 2020, Jung et al. [22] proposed an algorithm called Deep Vision (DeepVision) to verify the abnormal blink details of characters in videos from the perspective of blink period, number of repetitions, and blink time. After actual operation verification, the method can effectively detect 7 out of 8 kinds of fake videos. Yang et al. [23] proposed a detection method based on detecting inconsistent head poses in videos in 2019. This method can reveal the wrong information about 3D head poses in fake videos, to identify the original video. of authenticity. Almost during the same period, Li and Lyu [24] proposed a method to expose deepfake videos by detecting facial distortion details. Since deepfake technology can only generate images of limited resolution that need to be further distorted to match the original faces in the original video, the method does not require deep fake videos as examples of negative training but instead generates fake videos by itself, thus greatly saving the workload of training. In addition, Qi et al. [25] first proposed identifying deepfake videos from the perspective of heartbeat rhythm; Ciftci et al. [26] detected deepfake videos from biosignal residuals; Liu et al. [27] detect fake faces from skin texture details.

The other part of the detection work mainly starts from the time domain and frequency domain features of the video and uses the method of directly learning the overall image features by complex networks for authenticity identification. In 2020, Qian et al. [28] proposed a face forgery detection video method based on mining frequency perception clues and created a new type of face forgery frequency detection network (F3-Net), which uses two different but complementary frequency senses and clues to detect the authenticity of subtle forgery artifacts or compression errors. Finally, the actual test results are obtained. Since the face can be tampered partially or as a whole, Dang et al. [29] believed that the tampered spatial information may not be necessarily very important. Therefore in 2020, they proposed a method of adding an attention mechanism to the baseline network to detect the entire video frame to distinguish the authenticity of the video. The attention mechanism they proposed can be grafted into a variety of different neural networks and intuitively show the tampered part of the fake video frame image. In 2020, Li et al. [30] proposed a new type of fake video detection network and directly displayed the deepfake synthetic boundary by X-ray. After inputting the grayscale image of the video frame image, the network can display whether the grayscale image to be tested is spliced from two different pictures. If the image is forged, the splicing curve will be marked. Unfortunately, the preprocessing of the dataset is tedious and the workload is large. In the same year, Bonettini et al. [31] proposed a new network-based method for detecting deep fake videos based on EfficientNet-B4. This method utilized end-to-end and Siamese training methods and added a new attention mechanism to improve the baseline network. The face pixel position that has a great influence on network training parameters in the detection process is intuitively displayed, which provides a new direction for the detection of fake videos. In addition, Nguyen et al. [32] used a novel capsule network to detect deepfake videos; Li et al. [33] proposed a deepfake detection method using multi-instance learning; Hashmi et al. [34] created a Conv-LSTM hybrid architecture for deepfake video detection; Frank et al. [35] started with frequency analysis to identify fake images.

The article "Deepfake Video Detection Based on EfficientNet-V2 Network" was published in 2022. Journal: Comput Intell Neurosci.

With the continuous deepening of research on deepfake videos, many new detection methods with high efficiency and high accuracy have emerged in the academic world recently. Zhang et al. [36] invented a pseudofeature extraction technology for face exchange images based on deep learning and error level analysis. They used the ELA method to improve the efficiency of the CNN model and then accurately extracted pseudofeatures with different compression ratios. Chugh et al. [37] argued that audio-visual desynchronization can be used as a basis for detecting deepfake videos and proposed Modality Dissonance Scores (MDSs) based on modality consistency to determine real and fake videos, which can eventually determine precisely which frames have been faked. Cozzolino et al. [38] learned temporal facial features through metric learning and an adversarial training strategy and came to the conclusion that only training on real videos can achieve high detection accuracy and good generalization. Zhao et al. [39] regarded the deep fake detection problem as a fine-grained classification problem and proposed a multiattention deep fake detection method, which was verified to be significantly better than ordinary binary classifiers. Sun et al. [40] proposed a novel detection network named LRNet, which utilizes precise geometric features to improve the efficiency and robustness of deepfake video detection.

The article "Deepfake Video Detection Based on EfficientNet-V2 Network" was published in 2022. Journal: Comput Intell Neurosci.

## 3. Proposed Method

In this subsection, we mainly introduce the two main work points of the paper. The first work point is the collection of the datasets and the preprocessing process of the datasets; the second work point is the improvement and optimization process of the EfficientNet-V2 network.

### 3.1. Dataset Collection and Preprocessing

If deep learning is to be used to train new networks, a good and convincing dataset is essential. Through preliminary literature research and preparation, we have collected many large-scale public datasets about fake face datasets from the Internet. For convenience, we organize their basic information in the form of a table, as shown in Table 1.

In recent years, researchers have made great efforts to detect deepfake videos. With the advancement of detection technology, the demand for data is also increasing year by year, and the corresponding deepfake video datasets are constantly being updated. Considering various factors, we finally choose to use the most convincing FaceForensics++ fake face video dataset and the newly released FFIW_10K_ fake face video dataset (shown in bold in Table 1) for training and verification of the network model.

After selecting the appropriate dataset, which is convenient for the training and verification of the network, we convert the video-level dataset into a picture-level dataset by preprocessing the dataset. The entire workflow is shown in Figure 1. First, the authentic and fake videos are stored in two folders, respectively, and the authentic and fake videos are marked. The videos in the two folders are, respectively, processed by video framing. In order to improve the diversity and richness of the image dataset, we choose to extract a frame image every 30 frames when the video is divided into frames. In order to enable the network to fully learn the faces and their surrounding parts in the real and fake pictures, face recognition and cropping work are performed on the video frame images. Using the face 68 feature point detection script in Dlib, all faces in the picture can be accurately identified. In order to extract the surrounding parts, we expand the size of the crop so that we can extract several real and fake face pictures according to the number of faces in the video frame. Due to some errors in the script, the extracted pictures need to be screened by us to delete nonface pictures (patterns similar to human faces on clothes or walls), blurred face pictures, and incomplete face pictures, so as to keep clear and complete squares real and fake face pictures. Finally, the processed real and fake face pictures are uniformly scaled and numbered in turn, respectively, saved to the real face pictures and forged face pictures in two folders. So far, all the dataset preprocessing work is completed.

The article "Deepfake Video Detection Based on EfficientNet-V2 Network" was published in 2022. Journal: Comput Intell Neurosci.

The dataset preprocessing is performed on the FaceForensics++ fake face video dataset and the FFIW_10K_ fake face video dataset, respectively. According to the research requirements of this topic, 20K real face pictures and 20K fake face pictures are obtained from the two datasets, as shown in Figures 2 and 3. In order to explore the improved deep learning network model separately, we did not merge the datasets. In the later stage, the two datasets will be trained and verified separately, and finally, the original video will be detected.

### 3.2. EfficientNet-V2 Network

The multidimensional mixed model scaling method (EfficientNet series network) proposed by Google in 2019 has attracted extensive attention in the academic community. In order to explore a model scaling method that takes both speed and accuracy into account, the EfficientNet series network that simultaneously scales the three dimensions of network depth, network width, and image resolution is first proposed.

As shown in Figure 4, Figure 4(a) represents the baseline network model based on a convolutional neural network. The input is a three-channel color image with a width of W and a height of H. After the layer-by-layer convolution, the network could learn corresponding features in the picture; Figures 4(b)–4(d) represent three common methods of unilaterally scaling the network, respectively: Figure 4(b) is to improve the network from the perspective of the resolution of the input image and improve the network learning efficiency by proportionally enlarging or reducing the size of the input image; Figure 4(c) is to improve the network and improve network performance by changing the number of channels in each layer of the network; Figure 4(d) is to increase or decrease the number of network layers so that the network can learn more specific feature information and improve network efficiency.  Figure 4(e) shows that, in the EfficientNet network, the composite parameters are used to simultaneously perform the scaling of the above three dimensions, thereby improving the overall performance of the network.

The article "Deepfake Video Detection Based on EfficientNet-V2 Network" was published in 2022. Journal: Comput Intell Neurosci.

According to past experience, single-dimensional scaling is not as complicated as possible; it is also necessary to consider the resource occupation of the network and the learning rate of the network to find an appropriate scaling scale to maximize network efficiency.

The three-dimensional comprehensive scaling problem in the EfficientNet will be expressed in a formula. We call the entire convolutional network *J*, and its *n* convolutional layer can be regarded as the following function mapping:

(1) $$\begin{array}{c} Y_{i}=F_{i}\left(X_{i}\right). \end{array}$$

Among them, *Y*_*i*_ is the output tensor, *X*_*i*_ is the input tensor, and its dimension is set to 〈*H*_*i*_, *W*_*i*_, *C*_*i*_〉. For the convenience of expression, the Batch dimension in the tensor is omitted; then, the entire convolutional network *J*, composed of *k* convolutional layers, can be expressed as

(2) $$\begin{array}{c} J=F_{k}⊙\cdots ⊙F_{2}⊙F_{1}\left(X_{1}\right). \end{array}$$

In practical applications, multiple convolutional layers with the same structure are usually called a stage. For example, ResNet can be divided into 5 stages, and the convolutional layers in each stage have the same structure. In terms of stage, the convolutional network *J* can be expressed as

(3) $$\begin{array}{c} J=\underset{i=1\cdots n}{⊙}F_{i}^{L_{i}}\left(X_{\langle H_{i},W_{i},C_{i}\rangle }\right). \end{array}$$

Among them, the subscript *i* (from 1 to *n*) represents the sequence number of the stage, *F*_*i*_^*L*_*i*_^ represents the *i* Stage, which consists of the convolutional layer *F*_*i*_ repeated *L*_*i*_ times, and 〈*H*_*i*_, *W*_*i*_, *C*_*i*_〉 represents the dimension of the stage input tensor.

In order to reduce the search space, we fixed the basic structure of the network and only changed the three scaling dimensions mentioned above: the network depth (*L*_*i*_), the network width (*C*_*i*_), and the resolution of the input image (*H*_*i*_, *W*_*i*_). And we finally added a restriction; that is, the amplification of the network can only be multiplied by a constant magnification based on the initial network (EfficientNet-B0); then, we only need to optimize the corresponding constant magnification, to abstract the final mathematical model:

(4) $$\begin{array}{c} \begin{array}{c} \underset{\text{d},w,r}{\max}\text{Accuracy}\left(J\left(\text{d},w,r\right)\right)\\ s.t.\begin{array}{c} J\left(\text{d},w,r\right)=\underset{i=1\cdots n}{⊙}{\hat{F}}_{i}^{d\cdot {\hat{L}}_{i}}\left(X_{\begin{array}{c} \langle r\cdot {\hat{H}}_{i},r\cdot {\hat{W}}_{i},w\cdot {\hat{C}}_{i}\rangle \end{array}}\right)\\ \text{Memory}\left(J\right)\leq \text{Memory}\left(\text{target}\right)\\ \text{FLOPS}\left(J\right)\leq \text{FLOPS}\left(\text{target}\right) \end{array} \end{array}. \end{array}$$

Among them, d represents the network depth scaling factor, *w* represents the network width scaling factor, and *r* represents the input image resolution factor.

The article "Deepfake Video Detection Based on EfficientNet-V2 Network" was published in 2022. Journal: Comput Intell Neurosci.

According to continuous experiments, the EfficientNet network finally uses a mixed dimension scaling method, which uses *ϕ* mixing coefficient a to determine the magnification of the three dimensions:

(5) $$\begin{array}{c} \text{depth }d=\alpha^{\phi },\\ \text{width }w=\beta^{\phi },\\ \text{resolution }r=\gamma^{\phi },\\ s.t.\begin{array}{c} \alpha \cdot \beta^{2}\cdot \gamma^{2}\approx 2,\\ \alpha \geq 1,\beta \geq 1,\gamma \geq 1. \end{array} \end{array}$$

Among them, *α*, *β*, *γ* are constants obtained through the network search, and the mixing coefficient *ϕ* can be adjusted artificially. Considering that if the network depth is doubled, the corresponding calculation amount will be doubled, the network width or image resolution will be doubled, and the corresponding calculation amount will be quadrupled; that is, the computation amount (FLOPS) of the convolution operation is proportional to d, *w*^2^, *r*^2^, so the constraint in equation (5) has two square terms. Under this constraint, after setting the mixing coefficient *ϕ*, the computational complexity of the network will probably be 2^*ϕ*^ times that of the previous one.

The network is similar to the traditional convolutional neural network.  Table 2 shows the network framework of EfficientNet-B0. It can be seen that the network is divided into 9 stages in total. Stage1 is an ordinary convolutional layer with a convolution kernel size of 3 ∗ 3 and a stride of 2, which includes BN (Batch Normalization) and the Swish activation function. Stage 2–Stage 8 are all in repeated stacking of MBConv structures. The layers in the last column of the table indicate how many times the stage repeats the MBConv structure, while Stage 9 consists of an ordinary 1 ∗ 1 convolutional layer, an average pooling layer, and a fully connected layer, which contains BN and the Swish activation function. In the following table, each MBConv will be followed by a number 1 or 6, where 1 or 6 is the multiplication factor *n;* that is, the first 1 ∗ 1 convolutional layer in MBConv will expand the channels of the input feature matrix to *n* times, where *k*3 ∗ 3 or *k*5 ∗ 5 represents the size of the convolution kernel used by Depthwise Conv in MBConv. The channels represent the channels that output the feature matrix after passing through the stage.

(6) $$\begin{array}{c} f\left(x\right)=x\cdot \text{sigmoid}\left(\beta x\right). \end{array}$$

The expression of the Swish activation function is shown in formula (6), where *β* is a constant or set as a trainable parameter. The Swish activation function is lower bound, smooth, and nonmonotonic.

The article "Deepfake Video Detection Based on EfficientNet-V2 Network" was published in 2022. Journal: Comput Intell Neurosci.

The MBConv mentioned above is actually an improved version of the Inverted Residual Block. The Swish activation function is used in MBConv in the EfficientNet network, and SE (Squeeze and Excitation) module is added to each MBConv. The specific structure of MBConv is shown in Figure 5:

As it can be seen from the above figure, the MBConv structure is mainly composed of a 1 ∗ 1 ordinary convolution (dimension-raising effect, including BN and the Swish activation functions), a *k* ∗ *k* Depthwise Conv convolution (including BN and the Swish activation functions, *k* The value of is 3 or 5), a SE attention mechanism module, a 1 ∗ 1 ordinary convolution (dimension reduction, including BN), and a Dropout layer.

Regarding the shortcut connection, it exists if and only if the feature matrix of the MBConv structure has the same shape as the output feature matrix. The specific structure of a SE attention mechanism module is shown in Figure 6, which consists of a global average pooling layer and two fully connected layers. The number of nodes in the first fully connected layer is 1/4 of the input MBConv feature matrix channels, and the Swish activation function is used. The number of nodes in the second fully connected layer is equal to the channels of the feature matrix output by the Depthwise Conv layer, and the Sigmoid activation function is used.

The actual training and testing effect of the EfficientNet-V1 network, which is proud of its high efficiency, is not as efficient as the theory. Limited by the actual working conditions and working equipment, the speed of using Depthwise Convolutions in the shallow layer of the network will be very slow. In recent years of research, some people have proposed the Fused-MBConv structure to make better use of server accelerators. The Fused-MBConv structure is very simple; just replace the expansion con1 ∗ 1 and depthwise con3 ∗ 3 in the main branch of the original MBConv structure with an ordinary con3 ∗ 3 convolution, as shown in Figure 7. Replacing the MBConv structure with the Fused-MBConv structure can significantly improve the training speed. However, if all stages are replaced with Fused-MBConv, the number of parameters and FLOPS will increase significantly, and the training speed will also decrease.

Table 3 shows the model framework of EfficientNetV2-S. Compared with the model framework of EfficientNet-V1, the main differences are as follows:

- In addition to the MBConv module used in EfficientNet-V2, the Fused-MBConv module is also used (mainly used in shallow networks)
- The EfficientNet-V2 network will use a smaller expansion ratio (the first expand con1 ∗ 1 in MBConv or the first expand con3 ∗ 3 in Fused-MBConv), which is conducive to less memory access overhead;
- The EfficientNet-V2 network prefers to use a smaller kernel_size, and many 5 ∗ 5 kernel_size are used in EfficientNet-V1. It can be seen from Table 3 that the kernel_size used in the V2 network is all 3 ∗ 3. Since the receptive field of 3 ∗ 3 is smaller than that of 5 ∗ 5, it is necessary to stack more layers to increase the receptive field
- The EfficientNet-V2 network removes the last stage with a stride of 1 in the EfficientNet-V1 network because the number of EfficientNet-V1 parameters is too large and the access overhead is too large

The article "Deepfake Video Detection Based on EfficientNet-V2 Network" was published in 2022. Journal: Comput Intell Neurosci.

## 4. Experiments and Results

In this section, we mainly divide the discussion into two parts. The first part is using the EfficientNet-V2 network to train and test the preprocessed FF++ and FFIW_10K_ fake face datasets, recording the real-time Loss value and ACC accuracy of the training and test, and comparing the final training and test results with the existing ones. The detection accuracy of the datasets is compared, which objectively shows the superior performance of EfficientNet-V2 in detecting fake faces; The second part mainly describes the use of the trained network to detect the actual real and fake pictures as well as real and fake videos to achieve excellent visualization effects.

### 4.1. Dataset Training and Validation

In order to highlight the superior performance of the EfficientNet-V2 network we use on the FF++ dataset, we collect the detection accuracy ACC of the FF++ dataset in the current mainstream fake face detection network from various channels and sort them according to the accuracy, as shown in Table 4. According to Table 4, it can be clearly seen that the performance of the FF++ dataset on the XceptionNet network is particularly outstanding, and the detection accuracy can reach 96.36%. For the FFIW_10K_ dataset, due to the late release time, there is no official detection accuracy information for our reference. Based on the above criteria, we use the above two datasets to train and validate our network.

In order to explore the excellent performance of the improved new network, we train and verify the network and carry out analogy experiments from two perspectives of ACC value and Loss value. The experimental device is a Lenovo Legion R9000P2021H laptop with an 8-core 16-processor CPU from AMD Ryzen and an NVIDIA GeForce RTX 3060 6 GB graphics card. Training and validation are performed on two large-scale face authenticity datasets that have been preprocessed, respectively. The configuration parameters are as follows: the input image size is scaled to 224 ∗ 224, batch_size = 16, epochs = 50, freeze_layers (whether you need to freeze the network parameters of the backbone layer) = False, learn rate = 0.05, last learn rate = 0.01, and num_classes = 2. We randomly split the dataset into training and validation sets in a 9 : 1 ratio. The performance of the EfficientNet-V2 network on the FF++ dataset is shown in Figure 8, and the performance on FFIW_10K_ is shown in Figure 9. Among them, Figure (a) is the accuracy curve during training; Figure (b) is the accuracy curve during verification; Figure (c) is the Loss value decay curve during training; Figure (d) is the Loss value decay curve during validation.

The article "Deepfake Video Detection Based on EfficientNet-V2 Network" was published in 2022. Journal: Comput Intell Neurosci.

It can be clearly seen from the above two figures that after using the EfficientNet-V2 network to train 40K FF++ pictures and 40K FFIW_10K_ pictures 50 times, the ACC and Loss values tend to converge and stabilize. Relatively speaking, the real-time curve during training is smoother and more stable than the curve during validation. The validation accuracy on the FF++ and FFIW_10K_ datasets can reach about 97.9% and 93.0%, respectively, and the Loss value decays to about 0.053 and 0.183. After training and testing, the accuracy of the new network we used in detecting FF++ deep fake videos is 96.36% higher than that of XceptionNet, and it has also achieved very impressive detection results on the FFIW_10K_ dataset.

### 4.2. Actual Detection of Genuine and Fake Pictures and Videos

The main focus of this project is not only to explore the excellent performance of the new network in detecting genuine and fake pictures and videos but also to design a considerable effect of actually detecting genuine and fake pictures and videos. At present, using the excellent models that have been trained and verified, the real and fake pictures randomly extracted from the FF++ and FFIW_10K_ datasets are, respectively, detected, and the detection effect is shown in Figure 10.

As shown in Figure 10, we randomly take several authentic and fake images from the two datasets for actual detection. Figures 10(a) and 10(b) are real pictures in the FF++ dataset; Figures 10(c) and 10(d) are real pictures in the FFIW_10K_ dataset; Figures 10(e) and 10(f) are fake pictures in the FF++ dataset; Figures 10(g) and 10(h) are fake pictures in the FFIW_10K_ dataset. The input is a three-channel color image with a size of 300 ∗ 300, and the output is the original image with coordinates, the detected category (real or fake), and the predicted probability (output in the form of a percentage). It can be clearly seen that the predicted categories are consistent with the actual image categories, and the picture prediction probability is very high, indicating that the actual picture prediction effect is very good.

The article "Deepfake Video Detection Based on EfficientNet-V2 Network" was published in 2022. Journal: Comput Intell Neurosci.

On the basis that the network can efficiently predict the real and fake pictures, we have carried out in-depth research and exploration of the network predicting the testing effect of a whole video to be tested. Since each video to be tested is pieced together from frame-by-frame images, we decided to predict the video step by step. First, we split the video to be tested according to the unit of each frame, using facial recognition technology to select all identifiable clear face frames in each frame of an image. Next, we use the trained network to predict the authenticity of the face image selected by the frame and mark on the image frame after the prediction. After all the video frame image prediction was finished, we pieced together all the output images into a complete video according to the original timing sequence. Finally, a video can be output in which each frame of the image is authenticity detected and labeled. The specific video prediction process is shown in Figure 11.

In order to clearly observe the actual prediction effect of the video to be tested, we resplit the output video into video frame images to clearly observe the prediction effect of each frame, as shown in Figure 12, where the face is marked as a green box if it is recognized as real. If a fake face is identified, it is marked as a red box. At the same time, we have marked the corresponding discriminant probabilities after the discriminant. It is obvious that our network recognizes all video frame images of the video under test and can detect multiple faces in the image.

## 5. Conclusions

In this paper, we have produced a complete set of preprocessing schemes for real and fake video datasets and have demonstrated their feasibility through practical operations. Using FF++ and FFIW_10K_ large-scale fake face video datasets, a face image dataset of the order of 80K is produced. Moreover, the new EfficientNet-V2(S) network is used as the detection network for actual training and verification, and the entire training and verification process is recorded. As a result, the final trained network can achieve high-accuracy detection results. Aiming at the detection effect of actual images, we use the trained model to make actual predictions on the real and fake images randomly extracted from the two datasets and achieve a high prediction accuracy. From the image detection to the video detection, the video is split and detected and then reassembled, finally realizing the accurate detection of all clear faces in the video.

The article "Deepfake Video Detection Based on EfficientNet-V2 Network" was published in 2022. Journal: Comput Intell Neurosci.

In the future, we will continue to deepen the exploration and innovation of the baseline network. By improving the specific framework and details of the network. We can achieve higher detection accuracy. Based on ensuring efficient detection, we can improve the utilization of resources, shorten the time of training and actual testing, and improve detection efficiency. Besides, it is also one of the focuses of our future work to improve the generalization ability of the detection model as much as possible.

## Figures and Tables

**Figure 1:** Dataset preprocessing process.

**Figure 2:** FaceForensics++ dataset preprocessing result.

**Figure 3:** FFIW_10K_ dataset preprocessing result.

**Figure 4:** Model scaling comparison.

**Figure 5:** The specific structure of MBConv.

**Figure 6:** The specific structure of SE.

**Figure 7:** The specific structure of Fused-MBConv.

**Figure 8:** Training and validation performance on the FF++ dataset.

**Figure 9:** Training and validation performance on the FFIW_10K_ dataset.

**Figure 10:** The real and fake pictures detection renderings.

**Figure 11:** The video prediction flowchart.

**Figure 12:** The video frame images after prediction.

**Table 1:** Information about public datasets.

Name	Year	Real	Fake	Forgery methods
DeepFake-TIMIT [3]	2018	320	640	2
Deep fake detection [41]	2019	363	3068	5
**FaceForensics++** [13]	2019	1000	4000	4
DFDC [42]	2019	1131	4113	2
Celeb-DF [43]	2020	590	5639	1
DeeperForensics-1.0 [44]	2020	50000	10000	1
**FFIW**_**10K**_ [14]	2021	10000	10000	3

**Table 2:** EfficientNet-B0 network structure.

Stage	Operator	Resolution	Channels	Layers
1	Conv3 ∗ 3	224 ∗ 224	32	1
2	MBConv1, *k*3 ∗ 3	112 ∗ 112	16	1
3	MBConv6, *k*3 ∗ 3	112 ∗ 112	24	2
4	MBConv6, *k*3 ∗ 3	56 ∗ 56	40	2
5	MBConv6, *k*3 ∗ 3	28 ∗ 28	80	3
6	MBConv6, *k*5 ∗ 5	14 ∗ 14	112	3
7	MBConv6, *k*5 ∗ 5	14 ∗ 14	192	4
8	MBConv6, *k*3 ∗ 3	7 ∗ 7	320	1
9	Conv1 ∗ 1&Pooling&FC	7 ∗ 7	1280	1

**Table 3:** EfficientNetV2-S network structure.

Stage	Operator	Stride	Channels	Layers
1	Conv3 ∗ 3	2	24	1
2	Fused-MBConv1, *k*3 ∗ 3	1	24	2
3	Fused-MBConv4, *k*3 ∗ 3	2	48	4
4	Fused-MBConv4, *k*3 ∗ 3	2	64	4
5	MBConv4, *k*3 ∗ 3	2	128	6
6	MBConv6, *k*3 ∗ 3	1	160	9
7	MBConv6, *k*3 ∗ 3	2	256	15
8	Conv1 ∗ 1&Pooling&FC	—	1280	1

**Table 4:** The performance of the FF++ dataset on various networks.

Mainstream detection network	Accuracy (Acc) (%)
Xcept. full image	74.55
Steg. features	73.64
Bayar and Stamm	84.55
Cozzolino et al.	85.45
Rahmouni et al.	85.45
MesoNet	87.27
XceptionNet	96.36
**EfficientNet**	**97.90**

## Data Availability

The raw/processed data required to reproduce these findings cannot be shared at this time as the data also form part of an ongoing study.
